The article "Characterizing the Antitumor Effect of Coptis chinensis and Mume Fructus against Colorectal Cancer Based on Pharmacological Analysis" was published in 2022. Journal: Evid Based Complement Alternat Med.

# Characterizing the Antitumor Effect of *Coptis chinensis* and Mume Fructus against Colorectal Cancer Based on Pharmacological Analysis

**DOI:** 10.1155/2022/9061752

**Published:** 2022-06-23

**Authors:** RuiJiao Gao, Ying Lv

**Affiliations:** ^1^School of Traditional Chinese Medicine, Southern Medical University, Guangzhou 510515, China; ^2^Southern Medical University, Nanfang Hospital, Department of Ancient Traditional Chinese Medicine, Guangzhou 510610, China

## Abstract

Colorectal cancer (CRC) is the third most diagnosed cancer worldwide and is a significant cause of cancer-related deaths. Previous studies have observed that *Coptis chinensis* (CC) and Mume Fructus (MF) are effective against CRC, enteritis, and intestinal dysbiosis, but the chemical and pharmacological mechanisms remain poorly understood. In this study, we employed pharmacological network analysis to reveal mechanisms underlying the therapeutic effect of CC and MF against CRC. All compounds and targeted genes were obtained from the traditional Chinese medicine systems pharmacology database and analysis platform (TCMSP). Differentially expressed genes (DEGs) were identified based on GSE146587, GSE156720, and GSE184093 datasets. A protein-protein interaction (PPI) network was constructed to identify putative target genes of CC and MF. Ten key targeted genes were identified, including CCND1, ICAM1, IL1B, IL-6, MMP1, MMP3, MMP9, MYC, SERPINE1, and VEGFA. Among these genes, six (ICAM1, IL1B, IL-6, MMP1, MMP3, MMP9, and SERPINE1) were positively correlated with levels of effector memory CD4 T cells and natural killer T cells, and three (CCND1, MYC, and VEGFA) were negatively correlated with type 17 T helper cells and CD56dim natural killer cells. Molecular docking analysis showed that four compounds of CC and MF (kaempferol, oleanolic acid, quercetin, and ursolic acid) could affect CRC by interacting with target genes. Our study proved that pharmacological analysis could reliably assess the mechanism of traditional Chinese medicines for treating cancer.

## 1. Introduction

Colorectal cancer (CRC) is the third most common cancer worldwide, accounting for 10% of all cancers [1]. Unhealthy lifestyles and diet are risk factors for CRC [2], such as heavy drinking, tobacco smoking, and red or processed meat consumption, while supplementing calcium, whole grain, fiber, and milk products can diminish the risk [3]. Common symptoms of CRC include altered bowel habits, hematochezia, iron-deficiency anemia, weight loss, and stomachache [4]. Colonoscopy is considered the optimal method with the highest sensitivity and specificity among screening methods for CRC, which can detect and resect most cases of early CRC. However, colonoscopy is an invasive procedure that can cause patient discomfort and potential complications, limiting its widespread use in physical examinations [5].

Fortunately, the overall survival of advanced CRC has largely improved due to the advent of novel chemotherapeutic drugs and targeted therapies combining multidisciplinary therapeutics [6]. Nevertheless, these effective therapies have severe side effects, such as stomachache, constipation, and diarrhea. Therefore, new effective and safe therapeutics are still necessary. Traditional Chinese medicine (TCM) is a popular alternative to western medicine that has been applied in Asia for over 2000 years. The efficiency, abundant source, and the low incidence of side effects account for TCM's increasing popularity in other countries. In clinical cancer therapy, TCM involves treatment via prescriptions or serves as adjuvant therapy with conventional chemotherapy [7–9]. The methanol extracts of lead bioactive isolates of Dita bark are reportedly an effective source of antidepressants, anti-inflammatory drugs, and thrombolytic agents [10]. Besides, the methanol extracts of *Hedychium coronarium* (Zingiberaceae) have functions against oxidization, enzyme activity, and tumors [11], while those of *Rhamnus triquetra* (Wall.) are candidate components to develop new agents against multiple chronic diseases [12]. Additionally, the methanol extracts of *Psychotria calocarpa* leaves (MEPC) have neuropharmacological, analgesic, antidiarrheal, and antioxidization properties [13]; *Spirulina platensis* has great therapeutic potential against diseases involving inflammatory pain [14]. Cannabinoid receptors CB_1_ and CB_2_ and type 2 dopaminergic receptor (D_2_) exhibit antidepressive effects in models of depression and inflammation [15]. *Ophiorrhiza rugosa* var. prostrata is highly valued at the medicinal level in treating all kinds of pain conditions [16]. *Aglaonema hookerianum* Schott is recommended as an effective source of neuroprotective agents and as a candidate agent for sexual desire enhancement in cases of neural and sexual disorders [17]. *Tabebuia pallida* (Lindl.) Miers (*T. pallida*) have been reported to exert antitumor effects via induction of apoptosis [18]. Gynura possesses multiple pharmacological potentials against diabetes, oxidization, inflammation, bacterial infection, hypertension, and tumors [19]. *Andrographis paniculata* (Burm. f.) is capable of impeding invasive microorganisms and inhibiting biofilm formation [20]. Besides, *Lepidagathis hyalina* Nees are potential sources of antioxidants, cytotoxic agents, thrombolytic agents, antianxiety agents, and antidepressants [21]. Moreover, the seeds of *Syzygium fruticosum* (SF) have health-promoting effects and are the optimal candidate agents used to prevent degenerative diseases [22]. Green Tea Polyphenols are involved in immunoregulation and have antibacterial, antioxidant and anti-inflammatory activities, and it is used against diseases caused by the coronavirus [23]. The methanol extracts of *Molineria capitulata* have antioxidization, cytotoxicity, thrombolysis, anti-inflammation, and analgesic properties [24]. Last but not least, cannabinoids can be used as a source of new functional food ingredients and nutraceuticals, which are effective in treating and preventing gastrointestinal diseases [25]. Taken together, TCM herbs and their extracts play a huge role in pharmacological studies.

*Coptis chinensis* (CC) belongs to Ranunculaceae, composed of berberine, coptisine, *Coptis chinensis* Polysaccharide, quercetin, and so on [26]. CC has been widely used for treating bacillary dysentery, diabetes, pertussis, aphtha, eczema, and sore throat. Mume Fructus (MF) is the fruit of *Prunus mume* belonging to Rosaceae, generally cultivated in various regions in China, with the greatest output in the provinces south of the Yangtze River. Its major components include eugenol, dodecylic acid, ursolic acid, and quercetin. MF is commonly used for treating cough, bacillary dysentery, and sore throat in China. A combination of CC and MF is generally applied for treating ulcerative colitis, chronic diarrhea, and CRC. Although combined therapy of CC and MF is commonly used in clinical medicine, the active compounds and mechanism underlying their therapeutic effect against CRC remain unclear.

CC and MF combination is a multitarget and multicomponent formulation and is effective against CRC by regulating the intracellular molecular network. To investigate the specific mechanism of CC and MF in treating CRC, we applied bioinformatics and a multi-omics approach involving network pharmacology that has been established as important strategies for understanding TCM [27–30]. For example, Song et al. applied pharmacologic analysis to interpret the mechanism of triptolide in rheumatoid arthritis [31]. Zhang et al. revealed that Bushen Tiansui Formula positively affected cognitive improvement in Alzheimer's disease by using integrated analysis of pharmacology and serum metabolomics [32]. Yang et al. revealed the pharmacological mechanism of Rhizoma *Atractylodis macrocephalae* in treating gastritis based on pharmacological analysis [33]. The present study aimed to understand the mechanism of CC and MF treating CRC by using pharmacologic analysis and utilizing a series of CRC expression data from public databases. The workflow of the study is shown in Figure 1.

## 2. Materials and Methods

### 2.1. Analysis Based on the Pharmacologic Network

#### 2.1.1. Screening of Active Components in CC and MF

All compounds in CC and MF were obtained from the traditional Chinese medicines integrated database (TCMID, http://www.megabionet.org/tcmid/) [34]. The molecular weight (MW) of compounds is widely acknowledged to affect the efficiency of cell absorption; a high MW is difficult to absorb by cells, and compounds with WM between 180 and 500 are more suitable to be used as medicines, according to the Lipinski principle. Peroral drugs can function only after undergoing absorption, dispersion, metabolism, and excretion (ADME). During the process of ADME, drug-likeness (DL) is an important indicator for determining the active compounds [35]. Therefore, active compounds in CC and MF were included based on the screening criteria of MW ≤ 500 and DL ≥ 0.18.

#### 2.1.2. Constructing Drug-Target Interaction Networks

Protein targets of active compounds in CC and MF were acquired from TCMID and TCMSP databases. Cytoscape (v3.9) [36] was applied to construct CC/MF-active compounds-protein targets for visualizing the interaction between active compounds of CC/MF and their targets. In the network, drugs, compounds, and protein targets were all indicated as nodes, and their interactions were indicated as lines.

#### 2.1.3. Gene Set Enrichment Analysis on Drug Targets

To analyze gene ontology (GO) terms and Kyoto Encyclopedia of Genes and Genomes (KEGG) pathways of drug targets, the R package clusterProfiler (v4.0) [37] was employed. Functional terms were screened using the criteria count ≥2 and the expression analysis systematic explorer (EASE) score ≤0.05.

### 2.2. Analyzing Chip Data of CRC

#### 2.2.1. CRC Chip Data

CRC expression profiles of chip data were obtained from gene expression omnibus (GEO) database (https://www.ncbi.nlm.nih.gov/geo/). Three chips with CRC expression profiles were searched, including GSE156720, GSE146587, and GSE184093. The GSE156720 dataset based on the GPL26963 platform included the expression data of normal samples (*n* = 3) and CRC samples (*n* = 3). The GSE146587 dataset based on the GPL17077 platform included expression data of normal samples (*n* = 6) and stage III CRC samples (*n* = 6). The GSE184093 dataset based on the GPL20115 platform included data on normal samples (*n* = 9) and CRC samples (*n* = 9).

#### 2.2.2. Differential Analysis between Normal and Tumor Samples

The R package limma [38] was used to perform differential analysis between normal and tumor samples in the three datasets. A paired *t*-test was conducted to analyze data with normal distribution; otherwise, the Wilcoxon test was conducted to examine the significance of expression profiles between normal and tumor samples. *P* < 0.05 and |fold change (FC)| > 2 were used as screening criteria to identify differentially expressed genes (DEGs). Then, the pheatmap R package (v1.0.12) was employed to output the heatmap of hierarchical clustering and scatter plots to display the expression level.

#### 2.2.3. Identification of Key Drug Targets

The intersection between drug targets and DEGs identified in GSE cohorts was selected and analyzed in the STRING online tool (https://cn.string-db.org/). The results from STRING were visualized by Cytoscape (v3.9). The degree between each interaction was calculated, and top 10 genes with the highest degrees were considered key genes or drug targets.

### 2.3. Analysis of TCGA Data

#### 2.3.1. Acquisition of TCGA Data and Data Preprocessing

Samples of colorectal cancer were obtained from The Cancer Genome Atlas (TCGA) database (https://tcga-data.nci.nih.gov/). The TCGA-COAD dataset included 471 COAD samples and 41 normal samples, and the TCGA-READ dataset included 167 READ samples and 10 normal samples, where mRNA expression data and gene mutation data were included. The requirement for ethical approval was waivered by the ethics committee. The study met the standards of TCGA for publication. Genes in expression profiles were annotated based on Ensembl gene ID. Gene expression was transferred to log2 expression and normalized through NMM normalization in the limma package. The average expression was selected when multiple expression data of one gene were presented. Genes with averaged expression >1 were retained, and low expressed data was eliminated.

#### 2.3.2. Methodologies for Analyzing TCGA Data

Correlation analysis was assessed by the corrplot package (v0.92). Gene mutation analysis was conducted by maftools (v2.10.05).

#### 2.3.3. Characterizing Tumor Microenvironment (TME)

Single-sample gene set enrichment analysis (ssGSEA) [39] was used to calculate the proportion of immune cells based on a series of gene sets [40, 41]. To avoid deviation caused by tumor purity, the ESTIMATE algorithm was performed to adjust the enrichment score of immune cells [42]. A total of 24 cell types in TME were analyzed, including endothelial cells, eosinophils, fibroblasts, M0 macrophages, M1 macrophages, M2 macrophages, activated mast cells, resting mast cells, monocytes, neutrophils, memory B cells, naive B cells, activated dendritic cells, resting dendritic cells, activated NK cells, resting NK cells, plasma cells, activated CD4 memory T cells, resting CD4 memory T cells, naive CD4 T cells, CD8 T cells, follicular helper T cells, gamma delta T cells, and regulatory T cells. The expression of four immune checkpoints (PD-L1, CTLA4, PD-1, and PD-L2) was evaluated.

### 2.4. Molecular Docking for Active Compounds and Drug Targets

To confirm the interaction between key active compounds and protein targets, molecular docking was implemented. Proteins corresponding to drug targets related to CRC were obtained from protein data bank (PDB) (https://www.rcsb.org/pdb/home/home) [43]. Then, the AutoDocking Vina (v1.1.2) software [44, 45] was applied to modify the crystal structure, including adding hydrogen, removing hydrate and ligands, and optimizing and supplementing amino acids. A grid module was employed to implement molecular docking, and binding energy was used as a standard for evaluating the stability of molecular docking. The binding stability was strengthened by increasing the binding energy score.

## 3. Results

### 3.1. Analysis Based on the Pharmacologic Network

We obtained 87 active compounds of CC and MF from TCMSP and TCMID databases, with 48 belonging to CC and 40 to MF. One compound (quercetin) was found in both CC and MF. 56.25% (27/48) and 45.00% (18/40) of active compounds in CC and MF met the criteria of MW ≤ 500 and DL ≥ 0.18. Finally, 44 active compounds were retained for the following analysis. 196 protein targets of 44 active compounds were identified from the TCMSP database. A protein-protein interaction network was constructed based on 196 protein targets and 44 compounds, where 242 nodes were included with 2 drugs, 44 active compounds, and 196 protein targets (Figure 2(a)). Notably, four key compounds of CC and MF were identified with high degrees, including quercetin (Degree = 152), (R)-Canadine (Degree = 32), beta-sitosterol (Degree = 28), and magnoflorine (Degree = 24).

GO analysis revealed the top 10 enriched molecular function terms of CC and MF, including “response to xenobiotic stimulus,” “response to lipopolysaccharide,” “response to oxygen levels,” “response to decreased oxygen levels,” and “reactive oxygen species metabolic process” (Figure 2(b)). KEGG analysis showed that some tumor-related pathways were significantly enriched, such as “chemical carcinogenesis-receptor activation” and “IL-17 signaling pathway” (Figure 2(c)). The above results suggested that CC/MF formulation exhibited multi-target and multicomponent characteristics for treatment via regulating cellular networks.

### 3.2. Differential Analysis between Normal and CRC Samples

We compared expression data between normal and tumor samples in three datasets (GSE156720, GSE146587, and GSE184093) and identified a series of DEGs by comparing tumor samples to normal samples (Figures 3(a)–3(f)). In the GSE156720 dataset, 832 upregulated and 643 downregulated genes were detected. In the GSE146587 dataset, 1426 upregulated and 1385 downregulated genes were detected. Finally, in the GSE184093 dataset, 1040 upregulated and 1300 downregulated genes were detected. The intersection of DEGs among three datasets yielded 714 upregulated DEGs, and 706 downregulated DEGs in at least two datasets (Figures 3(g) and 3(h)).

Then we assessed the enriched GO terms and KEGG pathways of upregulated and downregulated DEGs, respectively. For upregulated genes, molecular function terms, such as “organelle fission,” “mitotic nuclear division,” “DNA replication,” and “regulation of mitotic cell cycle,” were significantly enriched (*P* < 0.05, Figure 3(i)). Immune-related pathways such as “cytokine-cytokine receptor interaction” and tumor-related pathways, such as “cell cycle,” “TNF signaling pathway,” and “p53 signaling pathway,” were significantly enriched (*P* < 0.05, Figure 3(j)), indicating that these upregulated genes were highly involved in tumor proliferation. For downregulated genes, “cellular divalent inorganic cation homeostasis,” “cellular hormone metabolic process,” and “regulation of metal ion transport” were significantly enriched (*P* < 0.05, Figure 3(k)). Enriched KEGG pathways in downregulated genes were related to cell metabolism, such as “cAMP signaling pathway,” “regulation of lipolysis in adipocytes,” and “pentose and glucuronate interconversions” (*P* < 0.05, Figure 3(l)).

### 3.3. Identifying Key Drug Targets Based on PPI Network Analysis

In the previous section, we identified DEGs that were CRC-associated genes. The intersection between potential target genes of CC/MF and CRC-associated genes yielded 28 target genes among upregulated DEGs and 15 target genes in downregulated genes (Figure 4(a)). Then these intersected genes were further analyzed by using the STRING online tool, and the degree of each node was calculated (Figure 4(b)). Top 10 target genes were determined as key drug targets, including CCND1, ICAM1 IL1B, IL-6, MMP1, MMP3, MMP9, MYC, SERPINE1, and VEGFA (Figure 4(c)).

### 3.4. Analyzing the Features of Key Genes in the TCGA-COAD Dataset

To verify the important role of these 10 key genes, we further characterized their features in two independent datasets (TCGA-COAD and TCGA-READ). We first evaluated them in the TCGA-COAD dataset. Ten key genes (drug targets) were significantly overexpressed in the TCGA-COAD dataset (Figure 4(d)), consistent with the result in GSE cohorts. Correlation analysis revealed positive correlations among these key genes, especially between MMP1 and MMP3, and IL-6 and MMP3 (R > 0.5). By analyzing TCGA mutant gene data, 56 out of 399 samples were found to have mutations in these 10 genes (Figure 4(f)). MMP9 exhibited the highest mutation with a mutation frequency of 5% (Figure 4(f)). Missense mutations accounted for most mutations, with C > T commonly observed.

Then we evaluated the relationship between key genes and TME by analyzing their correlation with immune checkpoints and immune cells. Analysis of the relationship with four important immune checkpoints (PD-L1, CTLA4, PD-1, and PD-L2) in TME showed that ICAM1 expression was strikingly associated with the expression of all four immune checkpoints (*P* < 0.01, Figure 4(g)). In addition, MMP1 and MMP9 were significantly correlated with CTLA4 and PD-L2 expression (*P* < 0.01). Furthermore, we calculated the enrichment score of 28 immune-related cells by ssGSEA and analyzed the correlation between the expression of key genes and the enrichment score of these cells (Figure 4(h)). The results showed that ICAM1 was positively correlated with most immune cells, especially natural killer T cells, natural killer cells, and memory CD8 T cells. Notably, only ICAM1 was correlated with activated CD8 T cells, indicating its critical interaction with T cell activation. 7 of 10 genes (ICAM1, IL1B, IL-6, MMP1, MMP3, MMP9, and SERPINE1) were positively correlated with memory CD8 T cells, memory CD4 T cells, regulatory T cells, natural killer T cells, and so on. Additionally, CCND1, MYC, and VEGFA were negatively correlated with most immune cells, which suggested that they may play an unfavorable role in immunotherapy.

### 3.5. Analyzing Molecular Features of Key Genes in the TCGA-READ Dataset

We validated 10 key genes in the TCGA-READ dataset and observed consistent results. Ten key genes were overexpressed in READ samples compared to normal expression, although 3 (IL1B, IL-6, and MMP9) showed no significant difference (Figure 5(a)). Stronger correlations among 10 key genes were observed in the TCGA-READ dataset compared to the TCGA-COAD dataset (Figures 5(b) and 4(e)). Mutational analysis showed that only 6 of 137 samples had mutations of 10 key genes (Figure 5(c)). ICAM1 exhibited the strongest correlation with immune checkpoints, especially PD-L2 and PD-1 (Figure 5(d)). According to the TCGA-COAD dataset results, 7 of 10 key genes were positively correlated with most immune cells, and ICAM1 exhibited the highest correlation (Figure 5(e)). VEGFA, MYC, and CCND1 were negatively correlated with most immune cells, suggesting that they may play a negative role in immunotherapy.

Overall, 10 key genes displayed similar performance in TCGA-COAD and TCGA-READ datasets. Few mutations were found in these 10 genes, indicating that these genes had high specificity in COAD and READ. In immune analysis, ICAM1, IL1B, IL-6, MMP1, MMP3, MMP9, and SERPINE1 all showed positive correlations with most immune cells, implying that CC and MF may exert an antitumor activity by interacting with these genes and immune cells, and thus control tumor development.

### 3.6. Molecular Docking between Active Compounds and Protein Targets

According to the interaction among drugs, compounds, and protein targets, we identified 10 key genes (protein targets) that were putative targets of active compounds. Then we applied the AutoDocking Vina software to conduct molecular docking between active compounds and protein targets (Figures 6(a)–6(j)). The predicted binding energy of 10 protein targets is shown in Table 1. Generally, low binding energy indicates stable binding and a high possibility of interaction. Quercetin was able to interact with all protein targets, and ursolic acid could interact with most protein targets (Figure 6). Among 10 protein targets, ICAM1 could interact with all four active compounds, including kaempferol, oleanolic acid, quercetin, and ursolic acid. These results demonstrated that CC and MF exert an antitumor effect against CRC via the interaction of these active compounds with key protein targets that could modulate TME.

## 4. Discussion

TCM holds an important place in Chinese pharmacological studies and clinical practice. In recent years, overwhelming evidence has substantiated that multiple TCM herbs and their extracts possess antitumor activities. Emodin is a type of anthraquinone derivative distributed in the roots and rhizosphere of diverse plants. It is a natural compound with antitumor activity, predominantly inhibiting cancer cell growth, and proliferation through weakening oncogenic growth signals, such as protein kinase B (AKT), mitogen-activated protein kinase (MAPK), HER-2, Wnt/-catenin, and phosphatidylinositol 3-kinase (PI3K) [46]. Coumarin and related compounds have high bioactivity and low toxicity. They are commonly used in treating prostate cancer, renal cell carcinoma (RCC), and leukemia, with the ability to induce apoptosis, autophagy and cell cycle arrest, antioxidization, and metastasis through activation of various signaling pathways in malignant cells. In the meantime, they can counter the side effects caused by chemotherapy [47, 48]. Multiple natural products have demonstrated antitumor activities by promoting cell apoptosis and inhibiting metastasis to slow cancer spread while reducing cancer cell proliferation and triggering death [49]. Some natural compounds have been shown to have the potential to act as aromatase inhibitors, and thus play a huge role in the treatment of gynecological tumors [50, 51]. TCM extracts also play important roles in studies on colorectal cancer. For example, cruciferous vegetables and their bioactive metabolites play antiviral and antibacterial roles via protecting cells from DNA damage and deactivating oncogenic substances. Additionally, they possess antitumor effects presenting with suppression of metastasis and generation of vessels that supply blood to the tumor through inducing cell apoptosis and inhibiting migration [52]. Flavonoid compounds, with antioxidant, anti-inflammatory, antibacterial, antifungal, and antitumor activities, are highly effective in alleviating clinical symptoms associated with diarrhea, mucositis, neuropathic pain, and chemotherapy for colorectal cancer [53].

In the present study, we applied pharmacologic network analysis to predict the possible mechanism of CC and MF in treating CRC. GSE cohorts were used to screen key genes, and TCGA datasets were used as independent datasets to validate key genes. Molecular docking was finally performed to confirm the molecular interaction between active compounds and key protein targets.

CC has been used to treat various inflammatory diseases for over a thousand years, to clear away heat and toxic materials and dry dampness, according to Chinese medicine theories. The medicinal value of CC was first documented in ShenMungHerbal, and over 32000 kinds of Chinese medicine formula, including CC in the form of pulvis, pills, decoction, and tablets, can treat diarrhea, emesis, abdominal distension, hyperpyrexia, toothache, diabetes, jaundice, and eczema [54]. Recent evidence suggests that CC has an extensive pharmacological activity against bacteria, viruses, hepatic steatosis, atherosclerosis, reperfusion injury after myocardial ischemia, diabetes, arrhythmia, hypertension, inflammation, and tumors [54, 55]. To date, over 120 compounds have been identified and extracted from CC; most compounds belong to alkaloids, followed by lignans, flavonoids, organic acids, and volatile oil. Interestingly, a study demonstrated that CC has a therapeutic effect against inflammatory bowel disease through inhibiting oxidative stress, protecting intestinal epithelium's barrier, alleviating pain, regulating T helper cells, and antimicrobial activity [56]. In addition, polysaccharides in CC can regulate immune responses related to the intestinal epithelium and intestinal microenvironment in an effective, dynamic, and dose-independent manner [57]. Moreover, epiberberine in CC is considered a potential drug for treating MKN-45-associated gastric cancer, targeting the p53-independent mitochondrial pathway [58].

MF has been used in traditional medicine for over 3000 years for treating fatigue, cough, headache, constipation, gastric diseases, and food poisoning. Growing evidence suggests that the major components of MF, including flavonoids, sterols, and organic acids, have multiple pharmacologic functions, such as bacteriostasis, antitumor activity, and regulating gut microbiota. Citric acid, chlorogenic acid, and neochlorogenic acid in MF can significantly alleviate cough and airway inflammation, inhibit the overproduction of mucus, and thus reduce chronic cough resulting from tobacco smoke in a guinea pig model [59]. Xing et al. illustrated that MF extracts could alleviate diarrhea caused by the combined treatment of lapatinib and Xeloda for breast cancer patients [60]. In addition, MF aqueous extracts can inhibit the expression of iNOS and COX-2, and the generation of PGE2, NO, and IL-6 induced by lipopolysaccharide (LPS) through blocking IkappaBalpha degradation and mitogen-activated protein kinase (MAPK) phosphorylation following with NF-kappaB activation [61].

Functional analysis of dysregulated genes in CRC samples showed that cell cycle-related processes “organelle fission,” “mitotic nuclear division,” “DNA replication,” and “regulation of mitotic cell cycle,” tumor-related pathways, such as “cytokine-cytokine receptor interaction,” and immune-related pathways, such as “Cell cycle,” “TNF signaling pathway,” and “p53 signaling pathway,” were significantly enriched, implying that these dysregulated pathways may be important mechanisms of CRC progression. We identified 10 key genes (CCND1, ICAM1, IL1B, IL-6, MMP1, MMP3, MMP9, MYC, SRTPINE1, and VEGFA) as putative targets of CC and MF during treatment against CRC. Some key genes have been reported to be associated with CRC development. In this regard, CCND1 has been documented to regulate the cell cycle in CRC tumorigenesis and development [62]. The MMP protein family promotes the malignancy of CRC cells through epithelial-mesenchymal transition (EMT) and Akt pathways [63]. Moreover, IL-6/IL-11 activates STAT3 in cancer-associated fibroblasts (CAFs) to promote CRC progression and poor prognosis [64]. Finally, a study found that the c-Myc/miR-27b-3p/ATG10 signaling pathway is involved in the drug resistance of chemotherapy in CRC [65].

Molecular docking demonstrated that the 10 protein targets could interact with four active compounds (kaempferol, oleanolic acid, quercetin, and ursolic acid) of CC and MF, which revealed the potential mechanism of CC and MF for treating CRC. Ten key genes identified in the study may serve as potential therapeutic targets for treating CRC. Furthermore, the study provides new directions for understanding CRC development based on CC and MF pharmacological network analysis. Taken together, our findings lay the groundwork for future pharmacological research and clinical applications, and provide an overview for the development of new drugs for colorectal cancer.

## 5. Conclusion

The present study combined network pharmacology, RNA sequencing, gene mutation, immune cell abundance, and molecular docking comprehensively discussed the mechanism underlying the therapeutic efficacy of the combination of CC with MF in CRC treatment, which involved suppression of inflammatory responses, cancer cell metabolism, and cell cycle process. Kaempferol, oleanolic acid, quercetin, and ursolic acid were identified as active compounds in CC and MF, while 10 key genes (including CCND1, ICAM1, IL1B, IL-6, MMP1, MMP3, MMP9, MYC, SRTPINE1, and VEGFA) were discovered as hub genes that played a mediating role in immunotherapy via triggering alterations of immune cells in the body, such as Natural killer T cell and memory CD8 T cell. During clinical practice, CC and MF are commonly used in combination to enhance immunity and inhibit cancer cell growth in cancer patients. The current study provided hitherto undocumented evidence of the mechanism of action of CC and MF in CRC treatment and broadened the therapeutic landscape for this patient population. However, our study still has some limitations. Indeed, no quantitative or experimental analysis of key active compounds was performed. In addition, only in silico research and limited CRC samples were used, warranting further validation in large-scale cell or animal experiments.

## Figures and Tables

**Figure 1:** The workflow of this study.

**Figure 2:** Identifying drug targets and analyzing their function based on the pharmacologic network.

**Figure 3:** DEG analysis on GSE cohorts. (a–f) Heatmaps and volcano plots of DEG expression in GSE156720 (a, b), GSE146587 (c, d), and GSE184093 (e, f) datasets. FC ≥ 2 and *P* < 0.05 were determined. (g, h) Venn plots of upregulated DEGs (g) and downregulated DEGs (h) in three datasets. (i, j) Bubble plots of top 10 enriched molecular function terms (i) and KEGG pathways (j) in upregulated DEGs. (k, l) Top 10 enriched molecular function terms (k) and KEGG pathways (l) in upregulated DEGs (*P* < 0.05).

**Figure 4:** Identifying key genes and molecular features of them in the TCGA-COAD dataset. (a) The Venn plot between DEGs identified from GSE cohorts and target genes of CC/MF. (b) A PPI network of 43 genes. (c) A PPI network of 10 key genes with top 10 degrees. (d) Expression of 10 key genes in normal and tumor samples. (e) A heatmap of correlation among 10 key genes. (f) A waterfall plot of top 10 mutated genes. (g) A heatmap of correlation between key genes and immune checkpoints. (h) A heatmap of correlation between key genes and immune cells. ^*∗*^*P* < 0.05, ^*∗∗*^*P* < 0.01, ^*∗∗∗*^*P* < 0.001, and ^*∗∗∗∗*^*P* < 0.0001.

**Figure 5:** Validation of 10 key genes in TCGA-READ dataset. (a) Expression of 10 key genes in the TCGA-READ dataset. (b) A heatmap of correlation among 10 key genes. (c) Waterfall plot of top 10 mutated genes. (d) A heatmap of correlation between key genes and immune checkpoints. (e) A heatmap of correlation between key genes and immune cells. ^*∗*^*P* < 0.05, ^*∗∗*^*P* < 0.01, ^*∗∗∗*^*P* < 0.001, and ^*∗∗∗∗*^*P* < 0.0001.

**Figure 6:** Molecular docking between active compounds and 10 protein targets. (a–j) Stimulation plots of interactions between 10 protein targets and active compounds. The green parts in A to J represent CCND1, ICAM1, IL1B, IL-6, MMP1, MMP3, MMP9, MYC, SRTPINE1, and VEGFA, respectively. (k) A pharmacologic network of CC/MF-active compounds-key genes.

**Table 1:** Results of molecular docking between active components and potential targets.

Targets	Binding energy (kcal/mol)			
	Kaempferol	Oleanolic acid	Quercetin	Ursolic acid
CCND1			−7.3	−8.0
ICAM1	−6.4	−7.1	−6.3	−7.0
IL1B			−7.5	−7.6
IL-6			−7.2	−7.4
MMP1	−8.7		−9.4	−7.2
MMP3			−9.4	−8.9
MMP9			−10.4	−8.2
MYC			−6.0	
SRTPINE1			−7.3	
VEGFA			−8.4	−8.6

## Data Availability

Data are available from the corresponding author upon request.
